The article "Platelet-Rich Plasma (PRP) in Breast Cancer Patients: An Application Analysis of 163 Sentinel Lymph Node Biopsies" was published in 2020. Journal: Biomed Res Int.

# Platelet-Rich Plasma (PRP) in Breast Cancer Patients: An Application Analysis of 163 Sentinel Lymph Node Biopsies

**DOI:** 10.1155/2020/3432987

**Published:** 2020-10-22

**Authors:** C. Eichler, C. Baucks, J. Üner, C. Pahmeyer, D. Ratiu, B. Gruettner, W. Malter, M. Warm

**Affiliations:** ^1^Department of Gynecology and Obstetrics, University of Cologne, Faculty of Medicine and University Hospital Cologne, Germany; ^2^Breast Cancer Center, Municipal Hospital Holweide, Cologne, Germany; ^3^Department of Radiology, Municipal Hospital Holweide, Cologne, Germany

## Abstract

**Introduction:**

Literature shows platelet-rich plasma (PRP) to improve overall outcomes in orthopedics, dermatology, ophthalmology, gynecology, and plastic surgery. Data on oncological patients is very limited. Only one publication is available on PRP in breast cancer patients. This work evaluated PRP in sentinel node biopsy procedures for breast cancer patients in terms of complication rates and oncological short-term follow-up.

**Methods:**

The evaluated PRP was ACP®, i.e., autologous conditioned plasma by Arthrex®. Between 2015 and 2018, 163 patients were offered to receive an ACP®/PRP injection in their lymph node biopsy site. Recruitment resulted in an approximate one-to-one ratio for analysis. Endpoints were major (revision) and minor (seroma, hematoma, and infection) complications rates as well as distant metastases, local recurrence, and overall survival. Median follow-up was 30 months.

**Results:**

Complication rates and oncological follow-up showed PRP to be applicable to use in a sentinel node biopsy scenario in breast cancer patients. There were 0 revisions in the ACP®/PRP group and 1.2% revisions in the control group (not significant). Oncological follow-up showed zero (0) distant metastases and local recurrences as well as a 100% 30-month overall survival.

**Conclusions:**

This is the first analysis of ACP®/PRP used in breast cancer patients in a sentinel node biopsy setting worldwide. PRP does not seem to increase rates of local recurrence within this 30-month follow-up time frame. Also, trend towards decreasing complication rates could be shown.

## 1. Introduction

Oncoplastic surgery is always aimed at improving overall surgical outcome. This research group recently published data regarding significantly improved patient satisfaction, postsurgical outcome, and complication rates on subcutaneous access devices in oncological patients when treated with platelet-rich plasma (PRP) [1]. In addition, literature shows improvement in overall outcomes in orthopedic surgery [2], conservative orthopedics [3–5], dermatology [6, 7], ophthalmology [8], gynecology [9], and plastic surgery. Complex wound management also found this product to be beneficial [10]. Especially the numerous positive results from the conservative PRP treatment of joints, justify a continuous investigation of the PRP issue. The overwhelming amount of available data is retrospective; this, however, leads to some meta-analyses on this topic comparing PRP to corticosteroids for mostly orthopedic procedures [11–13], again showing some benefit. Currently, there is no other data, apart from our previous work, towards a PRP application in breast cancer patients. This work will thus add a new area of interest, i.e., breast cancer patients that received PRP after a sentinel lymph node biopsy in the axilla.

Literature states PRP to not only contain platelets, but also growth factors such as platelet-derived growth factor (PDGF), transforming growth factor-*β* (TGF-*β*), basic fibroblast growth factor (bFGF), endothelial growth factor (EGF), and vascular endothelial growth factor (VEGF). These in turn improve wound healing although their possible oncological effect is entirely unclear [14, 15]. In order to decrease patient morbidity, we aimed to improve wound healing by instilling this PRP product subcutaneously after performing a single-incision sentinel lymph node biopsy in the axilla. Postoperative complication rates were to be evaluated. Major complications, such as revision surgeries, or minor complications, such as seroma and hematoma, may lead to subsequent interventions and increased patient morbidity. In addition, revision surgeries, seroma aspiration, etc. increase the financial burden on any health care system and should thus be avoided.

As a formal approach to the improvement of surgical technique, we require an evidence base. As randomized trials are difficult to fund, we nonetheless favor the adherence to the IDEAL framework for surgical innovation [16]. Three of the 4 stages were completed prior to this publication with the final stage, long-term study, being addressed within this work.

A fundamental problem in evaluating PRP products is patient subjectivity. Almost all patients subjectively feel better after receiving a PRP injection and or have knowledge of a PRP application. Thus, there will always be a subjective bias towards a positive outcome in a PRP treated collective when evaluated by questionnaire (i.e., pain and range of motion). This was shown in our previous work. Therefore, this evaluation focused on objective outcomes such as complication rates and recurrence only. The following questions were asked:

1. Is ACP®/PRP safe to use in a sentinel node biopsy scenario?
2. Is ACP®/PRP able to improve complication rates?
3. Is there an oncological risk for ACP®/PRP application regarding the short-term follow-up in oncological patients?

## 2. Patients and Methods

The PRP product evaluated in this trial was the autologous conditioned plasma system (ACP®—double syringe system) by Arthrex®. Thus, the terms PRP and ACP become interchangeable throughout this paper. The study was performed retrospectively at the Municipal Hospital Holweide, Breast Cancer Center, Cologne, Germany. Between these 2015 and 2018, patients were offered to receive ACP®/PRP injections in their lymph node biopsy site should the sentinel lymph node not be involved. As this choice in itself would introduce a bias, subjective outcome evaluations were omitted in this trial. All patients were offered the ACP®/PRP injections free of charge. This resulted in two cohorts of a total of 163 patients for retrospective analysis. The ACP®/PRP cohort included 82 patients, and the control cohort (no ACP®/PRP) included 81 patients. The one-to-one ratio was coincidental. No patients were excluded from this consecutive, retrospective analysis. There was no intent to form a one-to-one ratio. The initial overall goal was to stop recruitment when approximately 80 patients had received the ACP®/PRP product due to application cost.

In order to match both cohorts, group comparability had to be established with respect to the commonly known risk-factors for decreased wound healing such as age, BMI, type of surgery, prior chemotherapy, and smoking habits [17–19]. Once group comparability was established, the clinical outcome of this head-to-head analysis could be compared. Complication rates were divided into major and minor complication rates. Major complication rates, i.e., revision surgeries, were considered a severe adverse event as a significant increase in patient morbidity as well as patient discomfort and a financial burden to the medical system is introduced [17, 20, 21]. Minor complication rates include seroma, requiring and not requiring aspiration, hematoma, and infection. This type of complication rate analysis is commonly used in analyses of medical products in oncoplastic surgery. It allows a preliminary evaluation of the usefulness of any new product. As complication rates are generally very low, trial participation needs to be high in order to elucidate more than a trend and establish significance. This issue is often problematic as any product application and evaluation is limited by product costs.

### 2.1. Breast Surgery and Lymphadenectomy

All surgeries were performed by experienced breast surgeons, and gold standards were adhered to during all surgeries. All sentinel lymph node (SNL) biopsies were performed via a single incision. Preparation and identification of sentinel lymph nodes were done atraumatically, and a handheld gamma-detection probe was used to identify the target lymph node. Sentinel lymph node intraoperative frozen sections were performed for all patients in the ACP®/PRP only. All patients were node negative, i.e., no tumor cells were found in the lymph node, during surgery. After a full pathologic workup, some patients showed nodal involvement (12.2% ACP®/PRP vs. 17.3% control). Patients received either breast-conserving surgery (BCS) or mastectomy (MRM). The wound areas did not come into contact with the separate sentinel node biopsy area for any of the patients.

### 2.2. PRP Preparation and Application

The ACP® double syringe system (Arthrex, Naples, Florida, USA) was used during surgery. Procedures were followed as mandated by the manufacturer. Patient blood was extracted under sterile conditions during surgery via the port system or via a peripheral vein (see Figure 1). After centrifuge treatment, the double syringe system allowed the sterile transfer of the ACP®/PRP. It was then injected into the sentinel biopsy wound area subcutaneously, before a sterile dressing was applied.  Figure 2 shows several different separation stages of the ACP®/PRP.

### 2.3. Follow-Up

This low-risk cohort analysis was associated with a short-term follow-up. This is the first follow-up of any kind for ACP®/PRP in a low-risk oncological cohort. Evaluation included the endpoints: overall survival, local recurrence, and metastasis-free survival for a median follow-up of 30 months. Kaplan-Meier plots were not possible as zero events occurred.

### 2.4. Ethics Committee

Written informed consent was obtained from all patients. A copy of the written consent is available for review by the editor-in-chief of this journal. This study was conducted in accordance with institutional review board standard operating procedures. The application and production of a patient blood product were listed with Bezirksregierung Koeln, Dezernat 24: Öffentliche Gesundheit, Medizinische und Pharmazeutische Angelegenheiten.

An ethics committee approval/vote was obtained at the University of Cologne, Cologne, Germany, with ethics case number #20-1058.

### 2.5. Statistics

Statistical analysis was performed using the VassarStats® (Vassar College, Poughkeepsie, NY, USA) statistics program. Pearson's chi-squared tests and *t*-tests were used in order to evaluate significances when appropriate.

## 3. Results

In order to allow for intercohort comparability, it was important to establish equal distribution of risk factors.

The average age of the ACP®/PRP cohort was 59.7 ± 9.9 years and 62.5 ± 12 years in the control cohort (*p* = 0.13). The average BMI was 23.4 ± 3.4 kg/m^2^ for the ACP®/PRP cohort and 25.1 ± 5.2 kg/m^2^ for the control group. This difference is in slight, but significant, favor of the control cohort (*p* = 0.03). Results are shown in Table 1. 81.7% (*n* = 67) in the ACP®/PRP cohort received a breast-conserving surgery compared to 71.6% (*n* = 58) in the control cohort. The remaining patients had a mastectomy with or without implant reconstructions. All patients received separate, noncommunication incisions for the SNL biopsies. The differences in surgical procedures were not significant (*p* = 0.18). Smoking, prior chemotherapy, and prior or concomitant antihormone therapy did also not differ significantly. Note that prior radiation was omitted in the analysis since prior radiotherapy of the axilla would automatically prohibit a SNL biopsy. Thus, all above mentioned complication-associated risk factors were not significant (*p* = 0.69). Differences in grading, tumor size, hormone receptor status, and Her2 status were also not observed (see Table 2). Note that despite having a negative lymph node, i.e., no metastasis in the lymph node during intraoperative frozen section, 12.2% (*n* = 10, ACP®/PRP) and 17.2% (*n* = 14, control) of all patients showed some sort of nodal involvement when the complete pathological work-up was complete. This data included micrometastases. Nodal involvement did not exceed pN1a. Both cohorts do not differ. Therefore, regarding the oncological quality of the tumor, both cohorts were considered comparable.

### 3.1. Oncological Characteristics

All patients were early breast cancer patients. None of the patients had metastases. Table 2 shows a summary of patient characteristics. Cohorts did not differ in grading, immunohistochemistry, and/or involved lymph nodes. Due to this fact, administered chemotherapy and or radiation therapy did also not differ between these cohorts (see Table 1). There was no difference in BIRADS (Breast Imaging Reporting and Data System) classification regarding the initial tumor (all BIRADS 6). Regarding the lymph nodes, all ultrasound findings were negative; thus a sentinel node biopsy was required.

The key endpoints of this analysis, as seen in Table 3, show overall complications to occur in 21.9% (*n* = 18, ACP®/PRP) and 23.4% (*n* = 19, control) of all cases. Severe complications, i.e., revision surgeries did not occur in ACP®/PRP cohort and 1.2% (*n* = 1) needed a revision in the control cohort. Regarding minor complications, seroma requiring aspiration was found in 2.4% (*n* = 2, ACP®/PRP) and 3.7% (*n* = 3, control) of the cases. Seroma not requiring an aspiration was found in 19.5% (*n* = 16, ACP®/PRP) and 16% (*n* = 13, control) of the cases. Infections did not occur in either group. A trend favoring ACP®/PRP was seen for postsurgical hematoma with 0% (ACP®/PRP) vs. 2.5% (*n* = 2, control) of all cases (*p* = 0.25). Significance could not be reached. A 30-month follow-up for overall survival, local recurrence, and metastasis-free survival showed zero (*n* = 0) cases for both cohorts.

## 4. Discussion

After establishing initial comparability, we evaluated major and minor complication rates. As seen in Tables 1 and 2, comparability for both cohorts was given as risk factors were equal for both cohorts. Therefore, the subsequent endpoint analysis of major and minor complications could be performed. Overall, we found ACP®/PRP to have no disadvantages when applied.

As discussed in the introduction section, platelets contain a variety of growth factors, coagulation factors, adhesion molecules, cytokines, chemokines, and integrins. When activated, these entities are released causing an increase in concentration which is significantly higher than the baseline blood levels. This was thought to improve wound healing. However, a significant benefit could also not be established. Major complication rates in the control cohort, i.e., revision rates, were very low (1.2%, control) which means that in order to produce a significant difference, a study would have to vastly increase participant numbers. This is currently being done as ACP®/PRP application is continuously offered to all SNL patients at the investigation site. A follow-up publication will be attempted in the future. Minor complications, such as aspirated seroma and hematoma, numerically favor ACP®/PRP application although significance was also not reached. This could again be attributed to low patient numbers. Summarizing the complication data, it can be stated that ACP®/PRP was not able to produce a significant advantage in a SNL-biopsy scenario. Advantageous trends were observed; they do however require a follow-up trial.

In addition, this is the first short-term follow-up analysis for any ACP®/PRP data in oncological, specifically breast cancer, patients. Although the 30-month follow-up interval may be considered short, it is an important step towards establishing that ACP®/PRP in oncological patient does not seem to cause any concern. A 50-month (long-term) follow-up for the analysis of the treatment of subcutaneous venous access device is currently also being evaluated. Both of these results may begin to solidify our confidence in the safety of PRP in oncological patients.

Financially, the burden to the health care system is minimal. At approximately $50 cost for the ACP® double syringe system, costs are negligible. The subjective benefit of increased patient satisfaction, shown in our prior publication, itself should be enough to consider ACP® application. However, as objective complication rate analysis currently does not show a significant benefit, these authors consider ACP®/PRP application in a SNL scenario a possible and safe option, although we do not consider it a mandatory recommendation.

1. Is ACP®/PRP safe to use in a sentinel node biopsy scenario?

Preliminary data is promising. We were able to establish some data for ACP®/PRP use in oncological patients yielding no negative side effects.

(2) Is ACP®/PRP able to improve complication rates?

This remains somewhat unclear as the data is immature. We were able to show a slight trend towards improving hematoma and seroma rate. Significance could not be established.

(3) Is there an oncological risk for ACP®/PRP application regarding the short-term follow-up in oncological patients?

No. There were zero cases of recurrence and/or death in the 30-month follow-up. This product seems to be oncologically benign.

## 5. Trial Limitations

This work can be interpreted as hypothesis generating—a prospective and randomized trial would be needed to evaluate product impact onto overall short-term and long-term efficacy and safety. Within the scope of such a trial, a very homogenous patient group would have to be evaluated over a time period of ten to 15 years in order to evaluate short-term local and long-term distant recurrence risk.

## 6. Conclusion

This is the first analysis of ACP®/PRP used in breast cancer patients in a SNL biopsy setting worldwide. ACP®/PRP seems to be oncologically inert while displaying a trend towards decreasing complication rates. A zero cancer event risk in a 30-month follow-up was documented.

## Figures and Tables

**Figure 1:** Shown are the collection of peripheral blood into the double syringe system (a) as well as the placement of the double syringe system into a centrifuge (b). (c) Shows the subcutaneous application of the ACP/PRP product after SNL biopsy wound closure in the patient's left axilla.

**Figure 2:** Shown are the different stages of PRP preparation. The Arthrex ACP® double syringe system with whole blood (a) and after centrifugation (b). The double syringe allows the syphoning off of the PRP (c) which yields pure PRP, i.e., ACP (d). This product may now be injected.

**Table 1:** Shown are the patient characteristics for both cohorts.

	ACP/PRP		Control (no ACP/PRP)		*p* value
	No.	%	No.	%	
Patients (total *n* = 163)	82		81		
Breast-conserving therapy	67	81.7	58	71.6	
Mastectomy	15	18.3	23	28.4	0.18
Smoking^∗^	11	13.4	9	11.1	
Radiation^∗^	61	74.4	33	40.7	
Chemotherapy^∗^	18	22.0	22	27.2	
Hormone therapy^∗^	72	87.8	71	87.7	
Average age	59.7 ± 9.9		62.5 ± 12		0.13
Range	37-79		36-82		
Average BMI (kg/m^2^)^∗^	23.4 ± 3.4		25.1 ± 5.2		0.03
Range	17.6-35		17.9-40.5		
Postmenopausal	53	64.6	56	69.1	

^∗^All percentage data was calculated excluding the missing data (smoking: ACP *n* = 67, no ACP *n* = 71; Rtx: ACP *n* = 73, no ACP *n* = 73; Ctx: ACP *n* = 78, no ACP *n* = 74; hormone therapy: ACP *n* = 80, no ACP *n* = 79; BMI: ACP *n* = 66, no ACP *n* = 71).

**Table 2:** Documentation on tumor size and grading could not be procured for all cases due to the retrospective nature of this work. No patients were excluded.

	ACP/PRP		Control (no ACP/PRP)		*p* value
	No.	%	No.	%	
Patients	82		81		
Metastatis in SNL	10	12.2	14	17.3	0.3594
Tumor size^∗^
Tis	3	3.7	4	4.9	
T1	57	69.5	41	50.6	
T2	21	25.6	30	37.0	
T3	0		3	3.7	0.607
Grading^∗^
G1	15	18.3	17	21.0	
G2	49	59.8	46	56.8	
G3	11	13.4	18	22.2	0.7943
Hormone receptor status
Positive	72	87.8	72	88.9	
Negative	10	12.2	9	11.1	0.0037
HER2/neu
Positive	54	65.9	35	43.2	
Negative	28	34.1	46	56.8	0.0037

^∗^All percentage data was calculated excluding the missing data (tumor size: ACP *n* = 81, no ACP *n* = 67; grading: ACP *n* = 75, no ACP *n* = 81).

**Table 3:** Shown are the major and minor complication rates for both cohorts.

	ACP/PRP		Control (no ACP/PRP)		*p* value
Patients	82		81		
SLN removal via separate incision^∗∗∗^	75	91.5	45	55.6	
SNL removal via existing incision^∗∗∗^	7	8.5	36	44.4	<.0001
Total^∗^	18	21.9	19	23.4	
Major^∗^
Revision surgery	0		1	1.2	0.5
Minor^∗^
Seroma requiring aspiration	2	2.4	3	3.7	0.68
Seroma not requiring aspiration	16	19.5	13	16.0	0.68
Hematoma	0		2	2.5	0.25
Infection requiring antibiotics	0		0		

^∗^All percentage data was calculated excluding the missing data (ACP, *n* = 67 and no ACP, *n* = 73). ^∗∗∗^SNL: sentinel lymph node.

## Data Availability

All data is available upon request from the author.
